The article "The stability of quetiapine oral suspension compounded from commercially available tablets" was published in 2021. Journal: PLoS One.

# The stability of quetiapine oral suspension compounded from commercially available tablets

**DOI:** 10.1371/journal.pone.0255963

**Published:** 2021-08-10

**Authors:** Jennie Tran, Melissa A. Gervase, Jason Evans, Rebecca Deville, Xiaowei Dong

**Affiliations:** 1 Department of Pharmaceutical Sciences, University of North Texas Health Science Center, Fort Worth, Texas, United States of America; 2 Cook Children’s Medical Center at Fort Worth, Fort Worth, Texas, United States of America; ISF College of Pharmacy, Moga, Punjab, INDIA

## Abstract

Quetiapine fumarate (QF) is an atypical antipsychotic used off-label for the treatment of delirium in critically-ill infants and children. For the treatment of pediatric populations or patient populations with trouble swallowing tablets, an oral suspension would be an ideal dosage formulation. However, there are no liquid formulations of QF commercially available. Therefore, a compounded oral suspension prepared from the commercial QF tablets is widely used in clinical settings. The extemporaneous preparation of QF compounded oral suspension changes the formulation from a solid form to a liquid form. Thus, the stability of QF compounded oral suspension should be critically evaluated to guide pharmacists for administration and storage of QF compounded oral suspensions. However, the stability of the nonaqueous oral QF suspension was not measured. The objective of this study was to develop QF compounded oral suspensions at 10 mg/mL by using commercial QF tablets in two readily available aqueous vehicles (Ora-Sweet and Ora-Blend) and measure their stability at both room temperature and under refrigeration. Physical stability of the QF compounded suspensions were evaluated by appearance and odor. Chemical stability of the QF compounded suspensions were evaluated based on pH, degradation, drug content and the amount of the drug dissolved in the vehicles. An HPLC method was validated and used to evaluate QF compounded suspensions over 60 days. In addition to the total drug in the suspensions, the dissolved drug in the vehicles was also measured during the stability testing and evaluated as a stability parameter. Overall, QF suspension prepared in Ora-Blend was preferable, demonstrating a superior 60-day stability at both room temperature and refrigerated storage.

## Introduction

Delirium can be defined as acute changes in brain function that can result in sudden, severe confusion and disturbances in attention, developing directly from an underlying illness or its treatment [1,2]. Intensive care units (ICUs) have been shown to have high rates of delirium, occurring in 50–80% of mechanically ventilated adult patients [3]. ICU delirium is associated with prolonged hospitalizations, increased mortality, long-term cognitive impairment, and increased cost. Although under-recognized due to difficulty in developing appropriate assessment tools, ICU delirium can also occur in critically ill children at a rate of 12–65% [4]. Treatment of ICU delirium is multifactorial and includes both nonpharmacologic and pharmacologic interventions. There are currently no FDA approved medications for this indication; however, there is evidence that antipsychotics may be beneficial.

Quetiapine is a dibenzothiazepine atypical antipsychotic indicated for the treatment of schizophrenia and bipolar disorder in adolescents and adults [5,6]. Although the exact mechanism of action is unclear, quetiapine is an antagonist at multiple neurotransmitter receptors in the brain such as Serotonin 5-HT_1A_ and 5-HT_2_, dopamine D_1_ and D_2_, histamine H_1_, and adrenergic alpha_1_- and alpha_2_-receptors. Quetiapine is commonly used due to its short half-life allowing for rapid titration and favorable adverse effect profile. Case reports and small clinical studies have documented the successful use of quetiapine in the treatment of delirium in critically ill children and infants as young as 2 months of age [7–9].

Quetiapine is poorly water soluble and thus is marketed as its fumarate salt, Quetiapine Fumarate (QF), to improve its solubility. QF is currently only commercially available in the United States as immediate and extended-release tablets, limiting its application to treat ICU delirium in critically ill children [10]. A liquid dosage form is needed to be able to provide weight-based doses to infants and young children who are unable to swallow tablets. Therefore, the treatment of delirium in critically ill children and infants is relied on the extemporaneous preparation of a compounded oral QF suspension by pharmacists in clinical settings.

Although there is a published compounded protocol for 10 and 40 mg/mL compounded suspensions of QF, the formula was made in oil that was sticky, unpalatable, and generally disfavored [11]. Importantly, the stability of these nonaqueous oral QF suspensions was not measured. The extemporaneous preparation of QF compounded oral suspension changes the formulation from a solid form to a liquid form. Thus, the stability of QF compounded oral suspension should be critically evaluated to guide pharmacists for administration and storage of QF compounded oral suspension. The objective of this study was to develop QF compounded oral suspensions at 10 mg/mL using commercially available tablets in two readily available aqueous vehicles (Ora-Sweet and Ora-Blend) and measure their stability at both room temperature and under refrigeration. The stability of QF aqueous suspensions was analyzed by total drug content, the amount of the drug dissolved in selected vehicles, pH, visual appearance and odor in refrigerated and room temperature conditions for 60 days. We developed and validated an HPLC method for QF to study the stability of QF oral suspensions. The FDA drug stability guidelines were used to evaluate the data of stability for conclusion.

## Materials and methods

### Reagents and chemicals

A single lot of QF 400 mg tablet (Alkem, India) was used to conduct the stability testing. Ora-Blend and Ora-Sweet vehicles used in this study were obtained from Perrigo (Minneapolis, MN). Acetonitrile was purchased from Fisher Scientific Canada. Quetiapine standard, phosphoric acid and methanol was purchased from Sigma-Aldrich (MO, USA). Trimethylamine (TEA) was purchased from Janssen Pharmaceutical (Belgium). Water was purified using a Milli-Q Synthesis A10 system (Millipore, Etobicoke, ON, Canada).

### QF compounded suspension preparation from tablets

QF compounded suspensions (10 mg/mL) were prepared either in Ora-Blend or in Ora-Sweet. One QF 400 mg tablet was grinded to a fine powder by using a mortar and pestle. Two mL of propylene glycol was added to the mortar and pestle as a solvent and mixed to form a paste. After measuring 40 mL of the vehicle (Ora-Blend or Ora-Sweet) in a graduated cylinder, a small amount (2–5 mL) of the selected vehicle was added into the mortar and pestle and mixed until a uniform paste was formed. The vehicle was continually added, without using more than 50% of the total volume, until a pourable mixture was formed. This pourable mixture was transferred to a graduated plastic amber bottle. Using less than 15% of the total volume of the vehicle each time, the mortar and pestle was washed out into the amber bottle twice. The remaining amount of vehicle was then poured to quantum satis (Q.S.) into the plastic bottle until the final volume of 40 mL was achieved.

### HPLC method

The HPLC instrumentation (Waters, Milford, MA, USA) consisted of an Alliance 2695 Separation Module, equipped with a model 2487 wavelength ultraviolet detector. The column used was an Eclipse Plus 18 column (100 x 4.6 mm internal diameter, 3.5 mm particle size, Agilent, USA). The mobile phase A consisted of acetonitrile: methanol at 90:10 (v/v). The mobile phase B contained 200 μL of phosphoric acid and 500 μL TEA in 200 mL water. A flow rate of 0.8 mL/min was used for gradient elution. The elution started from 40% of mobile phase A for 0.5 min, then increased to 80% of mobile phase A within 4 min, maintained for 3 min and then changed to 40% of mobile phase A within 0.5 min and finally maintained at 40% of mobile phase A for 5 min. The injection volume was 20 μL. QF was monitored at a wavelength of 220 nm. QF peak had a retention time of about 5.9 min, and area of the peak was used to perform the quantification.

### HPLC method validation

The HPLC method was validated in terms of linearity, accuracy, precision, limit of detection (LOD), and limit of quantification (LOQ) according to the ICH guideline Q2(R1) [12]. The standard solutions were prepared by using an aliquot method. One hundred milligrams of QF were weighted and dissolved in 100 mL of methanol in a volumetric flask to prepare the stock solution. The stock solution was diluted with methanol to obtain the standard solutions at 1, 5, 10, 25, 50, and 100 μg/mL. The standard samples were injected in triplicate at three different concentrations (10, 25 and 50 μg/mL). The peak areas were used to calculate the mean and the % relative standard deviation (RSD) values. The calibration curve was constructed with six concentrations: 1, 5, 10, 25, 50 and 100 μg/mL. Each level of concentrations was injected in triplicate. LOD and LOQ were determined based on signal-to-noise ratios at 3 and 10 times, respectively. The accuracy was measured by the recovery of QF. The intra-day precision was tested with three injections per day for three days at three concentrations (10, 25, and 50 μg/mL). Force degradation samples prepared from stock solution were completed to evaluate the specificity of HPLC method, as well as predict and monitor the chemical degradation during the storage process. Forced degradation studies included four sets of samples: Set 1 (untreated), Set 2 (treated with 0.1 N HCl), Set 3 (treated with 0.1 N NaOH), and Set 4 (treated with 3% H_2_O_2_), which was conducted at 50 μg/mL of QF.

### Stability study designs

The stability of QF suspensions was tested for day 0, 7, 14, 30, and 60. After measured the stability at day 0, the preparations of the QF compounded suspensions (10 mg/mL) were stored in 30 amber PET bottles. The bottles were randomly divided to two even portions. Fifteen of the bottles was stored at monitored room temperature (22°C) and the other 15 were stored in a refrigerator (2°C). Three bottles were randomly pulled out and labeled #1, #2, and #3 to obtain three batches for each testing day and each temperature. On the testing day, the three batches that needed to be measured were taken back to room temperature, if stored in a refrigerator, and shaken very well before withdrew samples to obtain triplicate data. This design set the stability samples in three separate containers, which provided the independent triplicated measurement and storage.

### Physical tests of QF compounded suspensions during the storage

The physical tests were measured by changes in visual appearance, re-dispersibility, and odor. The changes in visual appearance included color, precipitation and solution clarity on the assigned testing days. The re-dispersibility was evaluated by homogeneousness of suspensions after manually shaking. The changes in odor were monitored by nose for the presence of unpleasant smell. The results were scored positive (+) for changes and negative (-) for no changes.

### Chemical tests of QF compounded suspensions during the storage

The chemical stability was evaluated in terms of pH, total QF drug content, the amount of the drug dissolved in the vehicle, and degradation. The pH of each sample was evaluated by a pH meter. To prepare samples for the measurement of total QF drug content, 1 mL of compounded oral suspension was drawn out from each plastic bottle and dissolved in 25 mL of a methanol/water (1:1, v/v) solution. After the mixture was vigorously vortexed and sonicated for 10 minutes, 1.5 mL of the mixture were transferred into a centrifuge tube and centrifuged at 14000 rpm for 5 min at 25°C. Then, 1 mL of the supernatant was collected and diluted with 10 mL methanol, and the solution was filtered with a 0.22 mm filter. The first 700 μL of the solution were discarded, and 180 μl of the solution were transferred into the HPLC vials for analysis.

To measure the amount of drug dissolved in the suspending vehicle, 1.5 mL of the compounded oral suspension were transferred into a centrifuge tube and centrifuged at 14,000 rpm for 5 min at 25°C. The supernatant was taken and centrifuged again to obtain the solution that contained the dissolved QF in the vehicle. The solution was diluted with 25 mL of a methanol/water (1:1, v/v) solution. Then, 1 mL of the mixture was further diluted with 10 mL of methanol and filtered with a 0.22 mm filter. The first 700 μL of the solution were discarded, and 180 μl of the solution were transferred into the HPLC vials for analysis. The degradation of QF suspensions was studied by monitoring the extra peaks in the HPLC chromatograms at the predetermined time points.

### Statistical analysis

Data are presented as mean ± standard deviation (SD). All experiments were at least repeated for three times, and the data were measured from three different batches.

## Results and discussion

### HPLC method development and validation

An accurate and precise analytical method is critical for the measurement of stability of drug formulations. HPLC separates impurities from drug substance through a column before a detector collects the signal of drug substance. Thus, it is widely used as an analytical method to measure drug content and degradations in a drug formulation. In this study, a new HPLC method using an Eclipse Plus 18 column was developed and validated for QF. Fumarate itself has absorption at 220 nm, which could interfere the absorption of quetiapine. Thus, the HPLC conditions need to separate fumarate and quetiapine. To maintain quetiapine at its neutral form and separate from fumarate, TEA and phosphoric acid were tested as a modifier of mobile phase. According to the results, phosphoric acid was selected as the modifier because of better separation and reproductivity compared to TEA. Gradient elution and a flow rate of 5 mL/min were used to obtain an optimal separation with adequate retention time.

The HPLC method was accurate over six injections for 10, 25, and 50 μg/mL (Table 1). The mean percentage of recovery for QF ranged from 102 to 111%. The linearity curve for QF was obtained with the correlation coefficient (R^2^) of 0.9995 in the concentration range of 1–100 μg/mL (Fig 1). The inter-day and intra-day precision measured the degree of reproducibility or repeatability of the analytical method under normal operating conditions are shown in Table 1. The RSD values for inter-day and intra-day precision were less than 2%. The LOD was detected at 0.5 μg/mL while the LOQ was determined at 1 μg/mL. The ingredients in both Ora-Blend and Oral-Sweet did not interfere with QF in the chromatograms. Thus, this HPLC method for QF is precise and accurate.

**Fig 1:** The linearity of QF standard solution in the HPLC method (n = 3).

**Table 1:** Accuracy and precision of the HPLC method (n = 6).

Parameter		Concentration (μg/mL)	Measured concentration (μg/mL)	Recovery% ^a^	RSD% ^b^
**Accuracy**		10	10.3 ± 0.1	103.7 ± 0.5	0.53
		25	26.9 ± 0.1	107.5 ± 0.4	0.36
		50	51.0 ± 1.0	102.0 ± 1.9	1.89
**Precision**	**Inter-day**	10	10.4 ± 0.1	103.9 ± 0.5	0.46
		25	26.9 ± 0.1	107.5 ± 0.4	0.36
		50	51.1 ± 0.7	102.2 ± 1.4	1.36
	**Intra-day**	10	11.0 ± 0.2	110.3 ± 2.0	1.82
		25	27.8 ± 0.3	111.1 ± 1.3	1.19
		50	50.9 ± 0.8	101.9 ± 1.6	1.61

a. Recovery% = Measured concentration/theoretical concentration x100%.

b. RSD% = SD/Mean x 100%.

### Forced degradation study

Force degradation samples are important to evaluate the specificity of HPLC method, predict and monitor the chemical degradation during the storage. It is known that QF mainly degrades under oxidative and hydrolytic conditions. Thus, the force degradation of QF was studied for acidic and basic hydrolyses and oxidation [13]. The results of forced degradation of QF are shown in Fig 2 for acidic hydrolysis, in Fig 3 for basic hydrolysis and in Fig 4 for oxidation. Retention time was a useful parameter to identify degradation products. After 24 hours, 84.9%, 33.1% and 11.5% of QF were degraded in 0.1N HCl, 0.1N NaOH and 3% H_2_O_2_, respectively. After 48 hours, 66.1% of QF were degraded in 0.1N NaOH and 100% of QF were degraded in both 0.1N HCl and 3% H_2_O_2_. The data demonstrate that QF was not stable in these testing conditions and the HPLC method was sensitive enough for detecting the reduced amounts of QF caused by the degradation.

**Fig 2:** Chromatograms of forced degradation samples of QF in 0.1N HCl for 24 hours and 48 hours.

**Fig 3:** Chromatograms of forced degradation samples of QF in 0.1N NaOH for 24 and 48 hours.

**Fig 4:** Chromatograms of forced degradation samples of QF in 3% H_2_O_2_ for 24 and 48 hours.

### Stability of QF compounded suspensions using Ora-Sweet and Ora-Blend

Limited by tablet sizes, the minimum dose of QF that can accurately be provided is 6.25 mg, which is one-quarter of a 25 mg QF tablet. The reported dosage range for QF in pediatric ICU delirium was 0.43 to 2.8 mg/kg/dose every 8 hours [14]. Therefore, 10 mg/mL oral suspensions were prepared in this study to provide a more accurate measurement to be used in the setting of pediatrics, especially in young infants and children.

Ora-Sweet and Ora-Blend are commonly used aqueous suspending vehicles in pharmacy because they are commercially ready-to-use. Both of them contains flavorants and preservatives. Thus, microbiological attributes are not needed to test for compounded suspensions when using these vehicles within their expiration dates.

Physical stability was monitored based on appearance and odor. The compounded samples were remained milky white (the appearance in Day 0 over 60 days without any abnormal colors. Additionally, the samples did not develop any unpleasant smell over 60 days. All samples were re-dispersible by manually shaking in the testing period of 60 days. The data indicate the physical stability of the tested QF nonaqueous suspensions over 60 days. The Ora-Sweet QF suspension tended to settle more over time than the Ora-Blend QF suspension, which could lead to a lack of dose uniformity in practice. This could be attributed to the formulation of the flavoring agents, as Ora-Sweet does not contain suspending agents in comparison to Ora-Blend. If using Ora-Sweet as the vehicle, vigorous shaking would be required to disperse the drug in the solution, making this a difficult formulation to use in clinical setting.

Chemical stability was monitored based on pH, degradation, drug content and dissolved QF. In clinical setting, QF compounded suspensions could be stored at room temperature (22°C) and in a refrigerator (2°C). Thus, both storage conditions were tested. The pHs of Ora-Sweet and Ora-Blend preparations were acidic with pH = 4.83±0.02 at Day 0. Over 60 days, the pH of both QF Ora-Sweet and QF Ora-Blend compounded suspensions rarely changed within a range of 4.78–4.89 in both storage conditions.

The targeted concentration in the QF compounded suspensions was 10 μg/mL. After the preparation, the measured concentrations of QF Ora-Sweet compounded suspension and QF Ora-Blend compounded suspension were 10.16±0.17 and 9.59±0.15, respectively. Thus, the concentrations of QF Ora-Sweet compounded suspension and QF Ora-Blend compounded suspension were 101.6% and 95.9% of the targeted QF concentration, respectively, which met the FDA criteria that the amount of preparation should be within 90–110% of the labeled amount. These results demonstrate that the QF compounding protocol in this study was reliable and able to prepare 10 mg/mL of QF suspension by using broken QF tablets.

According to the FDA guidance, significant change of a drug product is defined as a 5% change in drug content from its initial value [15]. In Tables 2 and 3, the measurements that were over 5% changes from their initial values are highlighted. According to the data, the drug contents for QF Ora-Sweet compounded suspension were less than 5% changes over 30 days at both temperatures and over 60 days at 2°C without degradation. However, the drug content for QF Ora-Sweet compounded suspension decreased over 6.6% and 26.3% for two batches out of three tested batches at room temperature, indicating instability at this condition that could be caused by hydrolysis. The drug contents for QF Ora-Blend compounded suspension were less than 5% changes over 60 days at both temperatures without degradation. Utilizing the goal of +/- 5% change, the data conclude that the QF in Ora-Blend preparation did not experience a significant change in drug content at 60 days in both room temperature and refrigeration.

**Table 2:** The changes of QF drug contents in QF Ora-Blend compounded suspension over 60 days at 2°C and 22°C (n = 3).

10 mg/mL	Sample number	Day 7	Day 14	Day 30	Day 60
	#1	-1.7	-1.8	-3.6	3.3
2 C	#2	1.8	-2.5	-4.2	0.7
	#3	0.0	-0.6	-3.6	3.6
	#1	0.9	0.8	-1.3	1.5
22C	#2	1.8	-1.7	-0.9	-0.9
	#3	1.7	0.3	-2.4	-0.1

Note: The changes are present at “- “for decreases and are bold for those over 5% compared to the initial value.

**Table 3:** The changes of QF drug contents in QF Ora-Sweet compounded suspension over 60 days at 2°C and 22°C (n = 3).

10 mg/mL	Sample number	Day 7	Day 14	Day 30	Day 60
	#1	-3.8	0.1	4.3	-3.2
2 C	#2	-3.3	2.8	1.7	4.2
	#3	-1.6	2.9	3.1	-4.8
	#1	0.2	0.7	1.7	3.6
22C	#2	4.5	1.7	0.7	**-26.3**
	#3	4.6	0.2	4.4	**-6.6**

Note: The changes are present at “-”for decreases and are bold for those over 5% compared to the initial value.

Since the QF tablet was crushed and further mixed into a liquid preparation, QF would be found as both dissolved and as suspended particles. The percentage of dissolved QF in the suspending vehicles could affect the bioavailability of QF. Thus, the amounts of QF dissolved in the compounded suspensions were monitored over 60 days at 22°C and 2°C. Tables 4 and 5, and Fig 5 indicate that storage conditions affected the amounts of dissolved QF in the suspensions. In refrigerated conditions, the percentage of dissolved QF in Ora-Blend decreased from 52.1% on day 0 to 42.5% by Day 14, and the percentage of dissolved QF in Ora-Sweet decreased from 48.0% on day 0 to 40.5% by Day 7. Room temperature storage also decreased the percentage of dissolved QF in Ora-Sweet from 48.0% on day 0 to 40.7% at Day 7. In contrast, the percentage of dissolved QF in Oral-Blend at 22°C did not have significant changes, as the concentrations remained above 50% through Day 60. Additionally, Fig 5 visually shows that QF in Ora-Blend stored at room temperature had both the highest amount of dissolved QF and also the most consistent level of dissolved QF over the entire 60 day testing period. Although sampling suspensions could generate the deviation on the measurements, it was clear that Oral-Blend at room temperature was better than other tested conditions in terms of keeping constant amounts of the dissolved QF. Thus, room temperature storage was preferable to keep the suspension with the same drug content as well as the dissolved QF from a given bottle over its 60 day storage time.

**Fig 5:** The percentage of dissolved QF in each suspension over 60 days at 2°C and 22°C (n = 3).

**Table 4:** The percentage of dissolved QF in QF Ora-Blend compounded suspension over 60 days at 2°C and 22°C (n = 3).

10 mg/mL	Sample number	Day 0	Day 7	Day 14	Day 30	Day 60
	#1	51.2	50.2	40.7	45.6	49.4
2 C	#2	52.6	52.3	43.6	44.6	49.4
	#3	52.7	55.4	43.2	44.7	49.3
	Average	52.1	52.6	42.5	45.0	49.4
	SD	0.8	2.6	1.6	0.5	0.1
	#1	51.2	51.8	55.7	51.7	53.3
22C	#2	52.6	54.6	54.4	51.8	52.7
	#3	52.7	53.7	52.7	50.5	51.5
	Average	52.1	53.4	54.3	51.3	52.5
	SD	0.8	1.4	1.5	0.8	0.9

**Table 5:** The percentage of dissolved QF in QF Ora-Sweet compounded suspension over 60 days at 2°C and 22°C (n = 3).

10 mg/mL	Sample number	Day 0	Day 7	Day 14	Day 30	Day 60
	#1	50.1	39.3	40.8	42.2	45.5
2 C	#2	47.6	40.6	41.3	42.9	45.5
	#3	46.4	41.6	43.1	41.9	44.7
	Average	48.0	40.5	41.8	42.4	45.2
	SD	1.9	1.2	1.2	0.5	0.5
	#1	50.1	40.7	41.1	42.0	46.2
22C	#2	47.6	40.9	42.1	43.3	46.9
	#3	46.4	40.4	41.0	43.8	47.0
	Average	48.0	40.7	41.4	43.0	46.7
	SD	1.9	0.3	0.6	0.9	0.5

## Conclusion

In this study, a reliable aqueous compounding formula for a 10 mg/mL suspension of QF was developed by using commercially available suspending agents, Ora-Sweet and Ora-Blend. An accurate and precise HPLC method was used to evaluate the stability of QF compounded suspensions over 60 days under both refrigerated and room temperature storage. Overall, the QF in Ora-Blend formulation showed better stability and better qualities than the QF in Ora-Sweet formulation. Room temperature storage of QF in Ora-Blend was shown to be the optimal storage condition for maintaining a consistent level of dissolved drug in the vehicle throughout the entire study period. The QF in Ora-Blend formulation demonstrated 60 day stability at both room temperature and refrigeration. However, it should be kept in mind that, although the study demonstrated the in vitro stability of compounded oral QF suspension, the in vivo performance of this compounded QF suspension is unknown. Since the data showed that the compounding process dissolved the parts of QF, it could be possible that the tablet, when taken as a whole, and the compounded suspension could have different oral absorption. Future studies are expected to compare in vivo absorption of tablets and compounded suspensions.
